# Multimodal Brain Image Fusion Based on Improved Rolling Guidance Filter and Wiener Filter

**DOI:** 10.1155/2022/5691099

**Published:** 2022-10-12

**Authors:** Hairui Lin, Yuhang Song, Hua Wang, Luoxin Xie, Dongfen Li, Guocheng Yang

**Affiliations:** ^1^College of Computer Science and Cyber Security (Oxford Brookes College), Chengdu University of Technology, Chengdu 610059, China; ^2^School of Mechanical and Electrical Engineering, Chengdu University of Technology, Chengdu 610059, China; ^3^Department of Electronic Information Engineering, Rizhao Polytechnic, Rizhao 276826, China

## Abstract

Medical image fusion technology can integrate complementary information from different modality medical images to provide a more complete and accurate description of the specific diagnosed object, which is very helpful for image-guided clinical diagnosis and treatment. This paper proposes an effective brain image fusion framework based on improved rolling guidance filter (IRGF). Firstly, input images are decomposed into base layers and detail layers using the IRGF and Wiener filter. Secondly, the visual saliency maps of the input image are computed by pixel-level saliency value, and the weight maps of detail layers are constructed by max-absolute strategy and are further smoothed with Gaussian filter, the purpose of which is to make the fused image appear more naturally and more suitable for human visual perception. Lastly, base layers are fused by visual saliency map based fusion rule and the corresponding weight maps from detail layers are fused by the weighted least squares optimization scheme. Experimental results testify that our method is superior to some state-of-the-art methods in both subjective and objective assessments.

## 1. Introduction

Medical image fusion from multiple imaging modalities, such as computed tomography (CT), magnetic resonance imaging (MRI) image, single photon emission computed tomography (SPECT) image, and positron emission tomography (PET) image, can provide a collective view of the lesion at a specific position of human body, which helps physicians to better understand the pathological conditions of the internal tissues and organs. Inherently, from any single modal image, it is difficult for the human eye to obtain complete and accurate information of the specific organ or tissue [1–3]. Multimodal medical image fusion techniques can integrate complementary information from multiple images acquired by different imaging sensors in the same target, so the expression of the fusion image in the same human body part is more accurate and reliable for diagnosis and assessment of medical problems.

Over the past two decades, many medical image fusion methods have been investigated at the pixel level [4–7]. Specially, multiscale transform- (MST-) based methods have been the hotspots of research and attracted the most widespread attention. For the MST based method, it is generally divided into three steps: decomposition, fusion, and reconstruction. To summarize, MST based method is more widely used, the process of which decomposes an image into the base layer and detail layers coefficients by applying selected transform tool. Further, a variety of fusion strategies are applied to combine different layer subimages and lastly achieves the fused results. Therefore, the selection of the MST tools and the fusion rules are two crucial factors and should be jointly considered for MST based image fusion.

In terms of image decomposition, some typical transform tools include, but are not limited to, Laplacian pyramid [8], complex wavelet transform [9], contourlet transform [10], nonsubsampled contourlet transform (NSCT) [11], shearlet transform (ST) [12], and nonsubsampled shearlet transform (NSST) [13]. With the flexible multiscale, multidirection, and shift invariant image decomposition function, the NSCT and NSST have manifested significant advantages and outstanding fusion performance compared with the other MST tools. Meanwhile, the conventional fusion rules are listed as follows: the averaging scheme, the max-absolute selection scheme, and weighted average scheme etc. In the past five years, researchers have proposed many image fusion algorithms based on NSCT and NSST. Zhu et al. [14] developed an NSCT-based medical image fusion method, in which, a phase congruency based fusion rule was introduced to merge the low-frequency component, and a local Laplacian energy rule was designed to fuse the high-frequency components. Wang et al. [15] proposed a medical image fusion method using the interscale and intrascale dependencies between multiscale image coefficients in the NSST domain. In their method, the dependencies of the NSST coefficients of the cross-scale and intersubbands are fully considered in the proposed fusion rule. In addition, pulse-coupled neural network (PCNN) model and MST based image fusion rule have been widely used in medical image fusion fields. Yin et al. [16] proposed a medical image fusion method with parameter-adaptive pulse-coupled neural network (PA-PCNN) in NSST domain. In their method, the PA-PCNN model and an energy based rule were used to fuse the high frequency and low-frequency coefficients, respectively.

Although many image fusion methods have achieved competitive performance, most approaches assume that the source images are noise-free, which may contain noise in actual tasks. For the fusion of noisy images, sparse representation- (SR-) based technique [7] is regarded as a good choice among numerous image fusion algorithms. To synchronously address the two problems of medical image fusion and denoising, recently, some joint image denoising and fusion algorithms based on SR have been proposed. Liu and Wang [17] proposed an adaptive SR method for image fusion and denoising. In this method, the appropriate dictionary is adaptively selected according to the image gradient features, and thus image fusion and denoising can be synchronously implemented. Kim et al. [18] designed a patch clustering-based dictionary learning method for multimodal image fusion. Although their method can effectively suppress noise generation, some important brightness information of source images cannot be well preserved in the fused images. In 2018, Li et al. [19] presented a joint medical image fusion, denoising, and enhancement method based on discriminative low-rank sparse dictionaries learning, to further improve the discriminative ability of the learned dictionaries. Afterwards, Li et al. [6] further developed a discriminative dictionary learning model to decompose input images into images coarse scale and fine scale components for detail-preserving noisy image fusion. In this scheme, an efficient multiple component dictionary learning model is formulated by integrating rank minimization into the low-rank component. However, this method is relatively complex and time-consuming. Li et al. [20] proposed a novel medical image fusion method based on the joint bilateral filter (JBF) and a gradient energy perception fusion rule, which decomposed a medical image into a structure layer with multilevel gradient and the energy layer containing rich intensity information by the JBF. Subsequently, Li et al. [21] proposed an image fusion method, i.e., joint image fusion and denoising via three-layer decomposition and SR, in which, the sparse reconstruct error parameter is adaptively designed according with the noise level, so as to realize the fusion and denoising for high-frequency components simultaneously.

With the rapid development of deep learning (DL) theory, meadical image fusion by DL is also one of the research focuses in recent years. Some DL based medical image fusion methods [22, 23] have emerged. Yu et al. presented a medical image fusion method based on convolutional neural networks (CNN) [24] for the first time in 2017, which achieved good results relative to the spatial domain and the transform domain. Subsequently, Liu et al. [23] also proposed a medical image fusion based on the convolutional sparse coding and morphological component analysis. However, this method has the flaw that the experiments are only tested on the gray scale medical images.

In recent years, multilevel edge-preserving filtering has been widely used in the field of image fusion. To gain better performance, researchers have proposed a variety of edge-preserving filters [25, 26] for recovering blurred image edges. However, most traditional edge-preserving filters only smooth details based on the contrast of the input image and do not take fully into account the spatial scale of input images. To address this issue, Zhang et al. [27] proposed a rolling guidance filter (RGF), which can smooth small structure information and include both scale aware and edge-preserving properties. Accordingly, many multiscale image fusion methods are introduced by applying RGF. Ma et al. [28] proposed a novel infrared and visible image fusion method that used the RGF and Gaussian filter to decompose input images into base layers and detail layers. Jian et al. [29] put forward an innovated image fusion method based on RGF and JBF filtering, in which RGF could remove small structures and recover the edges during the iterative process. Chen et al. [30] proposed a novel medical image fusion method based on RGF, and the method cannot only remain edge information but also maintain the energy of the source image.

In this paper, to resolve the synchronization problem of the fusion and denoising, we propose a medical image fusion algorithm based on improved RGF (IRGF), in which, in order to better extract the texture and edges of input images, the edge recovery process of images are repeatedly implemented using Wiener filter (WF) [31] to get the smoother images. Finally, the filtered outputs by IRGF and WF, base layers are fused by visual saliency map (VSM) based fusion rule, and the corresponding detail layers are fused by the weighted least squares (WLS) optimization scheme.

The main contributions of this paper are as follows:

(i) RGF is successfully modified to IRGF and used for brain image fusion based
  - on multiscale edge-preserving decomposition
(ii) a novel VSM based image fusion rule is introduced for base layers, which can improve the contrast and overall details of the resultant image
(iii) a WLS optimization scheme is introduced to merge the corresponding detail layers, thus the fused image appears more natural

The remaining subsections of this paper are organized as follows. In Section 2, we give a brief review of WF and IRGF. In Section 3, we will explain in detail the overall framework and fusion strategies. Qualitative and quantitative evaluation of experimental results are given in Section 4. Lastly, in Section 5, we conclude our work.

## 2. Related Works

### 2.1. Wiener Filter

The famous mathematician Norbert Wiener proposed a new linear filter in the 1940s, namely the Wiener filter (WF) [31]. This filter is also known as least mean squared error filter or least squares error filter. Conceptually, WF is an adaptive filter with the smallest mean squared error, and the output of the filter can be adjusted according to the local variance of input image. What is more, the larger the local variance, the stronger the smoothing effect of the filter [32–34]. Generally, WF is an adaptive filter that can calculate the mean and variance of a neighborhood, and it is also a low pass filter which can be applied to different contexts to restore noise-degraded signals. Thus, the optimal WF can be considered as one of the most fundamental noise reduction approaches, which has been confirmed in different forms and adopted in various applications. The definition of WF is defined as follows:

(1) $$\begin{array}{c} Wiener\left(I\right)=\frac{Boxfilter\left(I\right)}{N}+q*\left(I-\frac{Boxfilter\left(I^{2}\right)}{N}\right), \end{array}$$

where Boxfilter(·) is the filter for obtaining the difference of the matrix on the *X* and *Y* axes. *N* is the matrix obtained by putting an matrix of ones into Boxfilter(·). *I* is the input image matrix, and *I*^2^ is the square of the image matrix. *q* is the weight coefficient, which is defined as follows:

(2) $$\begin{array}{c} q=\frac{m}{m+eps}, \end{array}$$

(3) $$\begin{array}{c} m=\frac{Boxfilter\left(I^{2}\right)}{N}–\frac{Boxfilter\left(I\right)}{N}*\frac{Boxfilter\left(I\right)}{N}. \end{array}$$

where eps is the hyperparameter, and the value is set to 0.05.

### 2.2. Improved Rolling Guidance Filter

For the last decade, edge-preserving filters such as joint bilateral filter [35], guided filter [36], and weighted least squares filter [37]. have been widely applied in image fusion. Nevertheless, most of the conventional edge preserving filters rarely consider their spatial scales while smoothing small-scale structures of images. In order to preserve edge contents while smoothing image structures according to their scales, Zhang et al. [27] proposed a scale-aware edge-preserving filter in 2014, i.e., RGF, which includes both scale-aware and edge-preserving properties for image decomposition.

In RGF, a Gaussian filter is used to remove small structures, and a guided filter is used for edge recovery. In order to better remove small structures and highlight structure and edge contents of input images, in this work, we will improve the filtering way of the traditional RGF. The implementation process is modified to remove small structures through WF instead of Gaussian filter. Similar to the typical GRF, IRGF is also composed of two main steps, namely, small structure removal and edge recovery.

Firstly, small structure removal, we use a WF to smooth the input image, resulting in a smooth image without image details. Mathematically, the filtered image *G* from the input image *I* can be expressed as

(4) $$\begin{array}{c} \text{G}=\text{WienerFilter }\left(\text{I},\text{r},\lambda ,\text{N}\right), \end{array}$$

where *G* is the smoothed image; WienerFilter (∙) is a Wiener filtering operation, and *I* denotes the input image. *r* is the radius of template in the filter. In this paper, we set it to 3; *λ* is the regularization parameter; we set it to 0.01; *N* is calculated with a box filter for the size of each local patch.

Secondly, edge recovery, this step is iteratively implemented by using a joint filter, in which the guided filter is used as a joint filter to recover the edge details. It is an iterative process, i.e., the image recovered; *H*^*t*^ is iteratively updated; *H*^1^ is the image smoothed by the WF. The *H*^*t*+1^ is defined as follows:

(5) $$\begin{array}{c} H^{t+1}=GuidedFilter\;\left(H^{t},I,\sigma_{s},{\sigma_{r}}^{2}\right). \end{array}$$

Among them, GuidedFilter(·) is the Guided filtering operation; *H*^*t*^ is the smoothed image of the *t*-th iteration, and *t* is set as 4; *I* is the input source image,  *σ*_*s*_ is the standard deviation served as the scale parameter, and *σ*_*r*_^2^ is a regularization parameter which controls the range weight.

In general, IRGF is actually realized through the above two steps, and it can be simply written as

(6) $$\begin{array}{c} U=IRGF\left(I,\sigma_{S},\sigma_{r},T\right), \end{array}$$

where *U* represents the filtering output, and *T* is the iteration number which is set to 4 in this work.

In order to verify the superiority of the IRGF over RGF, we conduct the confirmatory experiment on two typical MRI and PET/SPECT image pairs, e.g. MRI-PET and MRI-SPECT fusions. For a fair comparison, we conduct the experiment using the same iterations (4 times) by applying IRGF and RGF.  Figure 1 provides a comparative example of the fused results produced by the IRGF and RGF based methods. For more intuitive comparison, some close ups are enlarged in the red regions and shown in Figure 1. By carefully observing the magnified version of the red regions marked of Figure 1, for the fused results produced by IRGF based method, we can see that the color information in the PET and SPECT images can better preserved and the edges are enhanced by considering the structural details of the MRI image. This experiment shows that, by applying IRGF, small-scale structures of an image are successfully removed according to their scales, while large-scale edges will be well retained. Simultaneously, using the WF to smooth the input image, all the edges of the filtered images are more blurred, which will be helpful to highlight large-scale edge details in the subsequent edge recovery.

### 2.3. Multiscale Decomposition Based on IRGF and WF

Accordingly, the proposed MSD based on IRGF and WF is formulated as follows:

(7) $$\begin{array}{c} u^{j}=IRGF\left(u^{j-1},{\sigma_{S}}^{j-1},\sigma_{r},T\right),\left(j=1,\cdots ,n–1\right), \end{array}$$

(8) $$\begin{array}{c} d^{j}=u^{j-1}-u^{j},\left(j=1,\cdots ,n–1\right), \end{array}$$

(9) $$\begin{array}{c} d^{j}=WienerFilter\left(u^{j-1},r,\lambda ,n\right),\left(j=n\right), \end{array}$$

(10) $$\begin{array}{c} d^{j}=u^{j-1}-u^{j},\left(j=n\right), \end{array}$$

where *u*^*j*^  is the *j-th* level filtered image; *d*^*j*^  denotes the *j-th* level detail layer, and *n* is the number of decomposition levels. The initial image *u*^0^ is the source image *I*.

Figure 2 provides the outputs obtained by repeatedly smoothing MRI image using IRGF, respectively, and the differences between adjacent images. It can be seen that, as shown in Figure 2, IRGF can effectively remove small-scale edges of input image while retain large-scale contents, and thus it can adequately extract detail features of the source images and preserve them well.

## 3. Proposed Method

The schematic diagram of the proposed fusion framework is shown in Figure 3. Firstly, taking for example the fusion of MRI and SPECT images, the source MRI image and the gray image obtained from SPECT by transformation are decomposed into base layer images *I*_*b*_^*MRI*^ and *I*_*b*_^*SPECT*^ and detail layer images *I*_*d*_^*MRI*^ and *I*_*d*_^*SPECT*^ using the IRGF an WF. Then, the base layers are merged based on VSM [38–40], namely, *VSM*_*MRI*_ and *VSM*_*SPECT*_, in terms of weighted average scheme aiming to obtain good contrast and more natural look in the final fused image. Next, the fusion of detail layers are conducted through the weighted least squares optimization scheme [28], in which the detail layers at different scales are defined by max-absolute strategy and subsequently smoothed by Gaussian filter.

After obtaining the fused subimages of the base layers and detail layers, the fused image *I*^*F*^ will be reconstructed by combing the fused base layer *I*_*B*_^*F*^ and the fused detail layers *I*_*D*_^*F*^. Lastly, the resultant image is reconstructed through the inverse transformation.

### 3.1. Fusion of Base Layers

In this section, we adopt a novel VSM-based weighted average scheme to fuse the base layer images. This technique has been widely used in many computer vision and computer graphics applications. For an image, the *VSM* of which can display perceptually salient visual structures or objects highlighting from their neighbors. As a result, the *VSMs* are usually used to describe the activity level measurement of source images for fusion tasks. In view of the fact that the *VSM* can reflect salient image features, we introduce the VSM to fuse the base layers, the calculation of which refers to the literatures [28, 38, 39]. Mathematically, it is defined as follows:

(11) $$\begin{array}{c} VSM\left(I=i\right)=Sal\left(i+1\right),i\in \left[0,255\right], \end{array}$$

(12) $$\begin{array}{c} Sal\left(j+1\right)=\overset{255}{\underset{i=0}{\sum }}Sal\left(j+1\right)+hist\left(i\right)*\left|j-i\right|,j\in \left[0,255\right], \end{array}$$

where *I* denotes the input image; *Sal*(·) is the salient pixel value of *j*; *hist*(*i*) is the *i*-th pixel value of the histogram computed by input image.

After the *VSM*_*A*_ and *VSM*_*B*_ are obtained, the base layer images and corresponding *VSMs* are performed by applying weighted average strategy, which is described as follows:

(13) $$\begin{array}{c} I_{B}^{F}=\left(\frac{1}{2}+\frac{{VSM}_{A}-{VSM}_{B}}{2}\right)*I_{b}^{A}+\left(\frac{1}{2}+\frac{{VSM}_{B}-{VSM}_{A}}{2}\right)*I_{b}^{B}, \end{array}$$

where *I*_*b*_^*A*^ and *I*_*b*_^*B*^ represent the base layers decomposed by input MRI/CT and SPECT/PET images, while *VSM*_*A*_ and *VSM*_*B*_ denote the *VSMs* of input MRI/CT and SPECT/PET images, respectively.

### 3.2. Fusion of Detail Layers

Basically, for the resultant image of MRI-SPECT/MRI-PET, the texture details mainly comes from MRI image while brightness information principally inherits SPECT/PET image. Since the characteristics that MRI/CT provides information with high-resolution soft tissue and SPECT/PET contains functional information with high intensity, it easily leads to loss of visually details and reduces the brightness of the fused image by using only the absolute maximum scheme. Therefore, it is necessary to make an improvement on the fusion rule which is usually used in the traditional method. With the above considerations, the WLS optimization scheme [41] is further introduced to fuse the detail layers, which is suitable for human visual perception. Firstly, the expression of the absolute maximum selection is as follows:

(14) $$\begin{array}{c} I_{abs}^{\max}=\left\{\begin{array}{cc} 1, & \left|d_{A}^{j}<d_{B}^{j}\right|\\ 0, & otherwise \end{array}\right.\left(j=1,2,\cdots ,n\right), \end{array}$$

where d_A_^*j*^ and *d*_*b*_^*j*^ are the *j-th* level detail layers decomposed by input MRI/CT and SPECT/PET images, respectively.

To make the fused image look more naturally, we use a Gaussian filter to smooth the image obtained by Equation (14). The Gaussian filtering is defined as follows:

(15) $$\begin{array}{c} G=Gaussion\left(I_{abs}^{\max},w\right), \end{array}$$

where Gaussion(·) is the Gaussian filtering; *w* is the size of filter, which we set to 3 in this paper.

Then, we figure out the detail layer images, the mathematical expression of which is described as follows:

(16) $$\begin{array}{c} I_{D}^{j}=\left(1-G\right)I_{d}^{1,j}+G\times I_{d}^{2,j}. \end{array}$$

Next, we use WLS to optimize the detail layer images obtained by Equation (16), and the mathematical expression is as follows:

(17) $$\begin{array}{c} I_{D}^{wls,j}=WLS\left(I_{h}^{j},I_{d}^{1,j},I_{d}^{2,j},\lambda \right), \end{array}$$

where *WLS*(·) is the calculation of weighted least squares value; *I*_*d*_ is a preliminary high-frequency image; *λ* is a hyperparameter, and its value is set to 0.01.

Finally, we will obtain the final detail layer image, which is expressed as follows:

(18) $$\begin{array}{c} I_{D}^{F,j}=I_{D}^{j}+I_{D}^{\text{wls},j},j=1,2,\cdots ,n. \end{array}$$

Finally, the fused image *I*^*F*^ can be reconstructed by combing the fused base layer *I*_*B*_^*F*^ and the fused detail layers *I*_*D*_^*F*^ as follows:

(19) $$\begin{array}{c} I^{F}=I_{B}^{F}+I_{D}^{F,\;j},j=1,2,\cdots ,n. \end{array}$$

## 4. Experimental Results and Analysis

The comparison experiments are conducted qualitatively and quantitatively on the publicly available dataset [42], which is a database website of the Harvard Medical School containing rich medical source images. Moreover, the runtime of different methods on three medical fusion tasks are provided and compared in the last experimental analysis.

### 4.1. Data Sets and Experimental Environment

To verify the superiority of the proposed method, six pairs of different types of brain images are used in our experiments, including multimodal images (CT-MRI, MRI-SPECT and MRI-PET). Furthermore, 30 pairs of MRI-SPECT images and 30 sets of MRI-PET images are selected to perform the experiment for quantitative comparison. All the test image pairs have the spatial resolution of 256 × 256 pixels, and they can be downloaded from http://www.med.harvard.edu/aanlib/home.html. This experiment is implemented on both AMD Radeon (TM) Vega 8 Graphics and 1.60 GHz Intel Core i5-8250 CPU using MATLAB.

### 4.2. Comparison Methods

In the experiments, we compared the proposed method with seven state-of-the-art fusion methods. These methods are as follows: fusion algorithm based on cross-bilateral filtering (CBF) [41], fusion algorithm based on neural networks (CNN) [43], image fusion based on sparse representation (ConvSR) [22], fusion algorithm based on dense network blocks and self-encoded structures (DenseFuse) [44], fusion Algorithm using a deep learning framework (VggML) [45], medical image fusion method based on unsupervised deep learning framework (EMFusion) [46], and a unified unsupervised image fusion network (U2Fusion) [47]. The source codes of these methods are all provided by their original authors, and all the parameters in the experiments are set as the default values.

### 4.3. Evaluation Metrics

For quantitative comparison, we select six metrics to evaluate the performance of the fused images, including spatial frequency (SF) [48], structural similarity (SSIM) [49], clarity measurement (CF) [50], extended spatial frequency (ESF) [51], average gradient (AG) [52] and visual information fidelity (VIF) [53]. Among them, SF, ESF, and CF are all image quality index that can effectively describe spatial features of an image, which indicates the overall clarity level of an image. SSIM measures the structural similarities between source images and the fused image. AG is also used to measure the clarity of the image and further analyze the texture details of the final image. VIF evaluates the percentages of visual information which is reserved between the source images and fused image. More detailed information can be provided in related references.

### 4.4. Parameters Analysis and Setting

It is necessary to investigate three free parameters in the proposed fusion mothod, namely, the hyperparameter *λ* of WF, the standard deviation *σ*_*s*_, and the regularization parameter *σ*_*r*_  of GuidedFilter in Equation (5). In Equation (4), the hyperparameter *λ* with the value range from 0.01 to 1 is used to control the trade-off between the saliency and abundance measurement results. When *λ* =0.01, the fused results cannot only preserve the abundant details in MRI image but also retain more color information in the SPECT/PET image. When *σ*_*s*_ increases, the regions with high pixel intensities are not preserved more completely. As a result, we set it to 0.01. For the parameter *σ*_*s*_ with the its range from 1 to 10 and the parameter *σ*_*r*_ with the range from 0.05 to 2, the experiment demonstrates that preserve both abundant details and color information at the same time when their values are set as 2 and 0.05. As a general rule, when we analyze one of the parameters, the other one will be fixed. Similar ways of discussing the impacts of multiple parameters have been widely adopted in some publications [36, 54, 55].

### 4.5. Visual Analysis

Figure 4 shows the MRI and CT images fused results produced by different methods. From these fusion results, we can easily see that the proposed scheme outperformed the other fusion methods, and the fused image has the best visual representation of both bone structure and soft tissue information for all eight methods. The fusion results of the other seven methods are shown in Figures 4(c–i), it can be seen that fused results of the VggML and U2Fusion methods not only have low contrast but also cannot clearly show the tissue characteristics of source MRI image. The fusion results produced by the CNN and EMFusion methods suffer from the oversaturated problem of intensity (see Figures 4(d) and 4(h)). Although the fusion images generated by the CBF, ConvSR and DenseFuse methods have better visual quality, there are artifacts at the edges of these images. Furthermore, by observing the red box regions, the proposed method introduces fewer artifacts and offers superior image quality in terms of resolution, brightness, and contrast. Figures 5(c–i) provide qualitative comparison results of the proposed method with seven competitors on the second pair of MRI and CT image fusion. It can be clearly seen that the final results on this pair of images are similar with the descriptions in Figure 4.

Figures 6 and 7 display the fused images of two pairs for MRI-SPECT image fusion using eight methods, respectively. It can be seen from Figure 6 that DenseFuse method produces low contrast and the color information is obviously distorted in the result image. The fusion image obtained by the U2Fusion method is low brightness and clarity. Although the VggML method gets better fusion performance, the contrast of the fused image is still not high, which may be caused by the average fusion rule. The CNN method introduces color distortion to a large extent. What is more, a lot of texture information in MRI image is lost, and there exists an overexposure phenomenon in the result of CNN. In contrast, the CBS, ConvSR, and EMFusion and our method have better visual effects and retain rich texture information in the source MRI image. The fused results of our method clearly have better contrast. Furthermore, compared with the red box regions which are enlarged, our method shows the optimal result in terms of color information, the contrast and texture details.

For MRI-PET images, we randomly select two pairs of images to show the effectiveness of the proposed method. As shown in Figures 8 and 9, the fused images of the CBF, ConvSR, and EMFusion decrease the brightness and contrast of the source images. Besides, the color information in the PET image is also distorted in the results generated by the aforementioned methods. The result obtained by CNN is overexposed, which seems to indicate that this method is not suitable for color medical images. As observed from Figure 8(d) and Figure 9(d), the edges in the MRI image are weakened to some extent in some competitors. For the U2Fusion method, both the background and the target area of the fused image appear dim, and the contrast is too low (see Figure 8(i) and Figure 9(i)). The DenseFuse method produces serious color distortion, which leads to the loss of a lot of functional information in PET image. Although the VggML method achieves relatively better visual effects, it still loses some details such as edges and textures. By comparison, the fusion results of our method are better than the others, in which the color information and texture details of the PET and MRI image are well enhanced and preserved. Besides, by comparing the enlarged regions marked of Figures 8–9, correspondingly. It can be clearly seen that the proposed method not only contains color information from the input PET image but also captures the texture details of the source MRI image.

### 4.6. Quantitative Analysis

In this work, six metrics are used to synthetically evaluate the performance of different fusion methods, which are, respectively, six metrics, i.e., SF, SSIM, CF, ESF, AG, and VIF. In theory, the bigger these metrics, the better the fusion result is. For better evaluation, three test datasets including 30 pairs of MRI-CT images, 30 pairs of MRI-SPECT images, and 30 pairs of MRI-PET images are selected to conduct experiments. The quantitative results obtained by eight different fusion methods on six metrics are shown in Table 1, Figures 10 and 11, respectively. Among them, the plotting for data visualization of the MRI-SPECT and MRI-PET fused results are shown in Figures 10 and 11. Note that the quantitative assessment values produced by different methods on six metrics are the average runtime in two graphs.

From Table 1, we notice that the values of CBF, CNN, ConvSR, and DenseFuse methods are slightly larger than ours in AG, SSIM, SF, and ESF evaluation metrics for MRT-CT fusion problems, but the fused results of the proposed method achieves the largest value in CF and VIF evaluation metrics. Furthermore, the values of our method, respectively, ranks second or third in SF, SSIM, ESF, and AG evaluation metrics. Overall, our algorithm achieved the excellent fusion performance for the MRI-CT fusion problems. Simultaneously, as shown in the quantitative results in Figure 10, we can observe that CBF is optimal on AG and suboptimal on SF, CF, and ESF. CNN is the third best on VIF, SF, DF, and ESF. ConvSR is suboptimal on AG. DenseFuse is suboptimal on VIF and ranks third on SSIM. EMFusion is suboptimal on MS-SSIM. Neither VggML nor U2Fusion has a good score on six metrics. Our results achieve the optimal results on SF, SSIM, DF, and ESF, with AG and VIF ranked third. The fused results on six metrics show that our method can well preserve the more valuable texture details in MRI/CT images and inherit the more color and brightness information in SPECT/PET images.

Similarly, the data visualization of the measurement values of MRI-PET image fusion by seven typical fusion algorithms and our methods is shown in Figure 11. It can be seen that our method achieves the optimal result on SF, ESF, AD, and CF and the pretty good results on SSIM and VIF. It shows that our fused result has comparative similarity with source images with less lost information. For the rest seven competitors, CBF ranks third on SF, CF, ESF, and AG. CNN is suboptimal on VIF. ConvSR is suboptimal on CF, ESF, and AG. DenseFuse is suboptimal on SSIM, the third on VIF. EMFusion is the second best on SF, and SSIM ranks third. Neither VggML nor U2Fusion achieves good results on six metrics. The quantitative comparison results indicate that our results can well retain the structural information in MRI images and the functional information in PET images by keeping high similarities with source images. Thus, it outperforms the other seven methods.

### 4.7. Execution Efficiency Comparison

The runtime comparison of different methods on three test datasets is reported in Table. It should be noted that the values in Table are the average execution time of different methods. As shown in Table 2, we can intuitively observe that the execution time of ConSR is the longest of all methods, and the execution time of CNN is also relatively long, slightly shorter than ConSR. By contrast, our fusion algorithm takes the shortest time and shows the optimal computational efficiency.

## 5. Conclusion

In this paper, we present an improved multimodal brain image fusion method based on multilevel edge-preserving filtering. Aiming to achieve a better scale separation while preserving information of image edges and reducing halos, the proposed method utilize the IRGF and Wiener filter to decompose source images into base and detail layers. Considering the conventional average fusion rule does not take full advantage of the residual information of base layers, the VSM-based weighted average strategy is referred to fuse base layers, which facilitates to achieve better overall appearance and high contrast in the final image. For the fusion rule of the detail layers, a novel WLS optimization scheme is introduced, which can overcome the limitation of conventional absolute maximum scheme by taking fully into account the characteristics of different modal medical images. In the meantime, this optimization process can effectively control the trade-off between the saliency and abundance measurement results of source images, and thus useful visual information and detail features can be better extracted and transferred into the resultant image while suppressing the noise from input images. Furthermore, the researches and applications of multimodal medical image fusion will be extended to the disease detection and diagnosis in the field of the precision medicine.

## Figures and Tables

**Figure 1:** Demonstration of the fused results obtained by RGF and IRGF, (a) and (b) and (f) and (g) are the source images. (c) and (h) are the fused results produced by applying RGF. (d) and (i) are the fused results produced by applying IRGF. (e) and (j) are the difference between the fused results produced by applying IRGF and RGF method.

**Figure 2:** (a) MRI image. (b), (c), and (c) and (e) are the output results obtained by 4 iterations of IRGF, respectively. (f), (g), (h), and (i) are the difference between (a) and (b), (b) and (c), (c) and (d), and (d) and (e). Notice that the data of (f), (g), (h), and (i) are multiplied by 5.

**Figure 3:** The schematic diagram of the proposed method.

**Figure 4:** Visual comparison of our method with seven state-of-the-art methods on the first pair of MRI and CT images.

**Figure 5:** Visual comparison of our method with seven state-of-the-art methods on the second pair of MRI and CT images.

**Figure 6:** Visual comparison of our method with seven state-of-the-art methods on the first pair of MRI and SPECT images.

**Figure 7:** Visual comparison of our method with seven state-of-the-art methods on the second pair of MRI and SPECT images.

**Figure 8:** Visual comparison of our method with seven state-of-the-art methods on the first pair of MRI and PET images.

**Figure 9:** Visual comparison of our method with seven state-of-the-art methods on the second pair of MRI and PET images.

**Figure 10:** Quantitative comparisons of six metrics, i.e., SF, SSIM, CF, ESF, AG, and VIF, on 30 test image pairs of MRI-SPECT images.

**Figure 11:** Quantitative comparisons of six metrics, i.e., SF, SSIM, CF, ESF, AG, and VIF, on 30 test image pairs of MRI-PET images.

**Table 1:** Quantitative evaluation for 30 pairs of MRI-CT fused images (bold: optimal).

Metrics	CBF	CNN	ConvSR	DenseFuse	VggML	EMFusion	U2Fusion	Ours
SF	34.22894	32.43961	**37.26421**	17.48996	20.15031	21.05623	18.64274	34.49011
SSIM	0.80156	**0.94015**	0.83193	0.31859	0.87559	0.88552	0.85524	0.92976
CF	9.69240	8.34933	8.84954	5.08303	5.38481	6.16628	6.10750	**9.78925**
ESF	0.03506	0.10140	0.04621	**0.50830**	0.43985	0.39173	0.46486	0.50422
AG	**8.30717**	7.05477	7.60956	4.27056	4.54141	5.32467	5.20886	8.03297
VIF	0.26443	0.45139	0.35529	0.05059	0.37849	0.40803	0.29462	**0.47872**

**Table 2:** Runtime comparison of different methods on three types of medical fusion tasks.

Method/type	CBF	CNN	ConvSR	DenseFuse	VggML	EMFusion	U2Fusion	Ours
MRI-CT	2.67	16.52	36.49	0.64	1.89	0.56	2.02	0.30
MRI-SPECT	3.73	17.57	30.87	4.09	4.02	0.42	1.82	0.30
MRI-PET	3.73	17.57	30.87	4.09	4.02	0.45	1.67	0.38

## Data Availability

(1) All the test image pairs can be downloaded from the Whole Brain Atlas dataset; they are publicly available at http://www.med.harvard.edu/AANLIB/home.html. (2) The codes of our work are, respectively, provided in the submitted program code. (i) the main program, code; (ii) the related functions called by the main program, code; (iii) the code of three comparative examples (Figure 1, Figure 2, Figure 3) using RGF and IRGF decomposition, code; (iv) quantitative comparisons of spect_evaluate, code; (v) quantitative comparisons of pet_evaluate, code; (vi) runtime of fusion on 30 pairs of MRI-SPECT images and code; (vii) runtime of fusion on 30 pairs of MRI-PET images, which is explained in detail. (3) Six metrics, i.e., SF, SSIM, CF, ESF, AG, and VIF and the results for the comparison were obtained from the source codes provided by the authors. All the parameters in the experiments are set to the default values. (4) The experiments are implemented on both AMD Radeon (TM) Vega 8 Graphics and 1.60 GHz Intel Core i5-8250 CPU using MATLAB. (5) The resultant images obtained by our method on 30 pairs of MRI-SPECT images and 30 pairs of MRI-PET images are provided as a supplementary material in “Data Availability” statement. (6) The data used to support the findings of this study are currently protected. Requests for data, (6/12 months) after publication of this article, will be considered by the first author or corresponding author.
